The article "Application Effect and Prognosis of High-Quality Nursing in the Whole Process of Nursing in Lung Cancer Surgery" was retracted in 2023. Reasons: signs of a paper mill; compromised peer review; unreliable results or conclusions.

# Application Effect and Prognosis of High-Quality Nursing in the Whole Process of Nursing in Lung Cancer Surgery

**DOI:** 10.1155/2022/9491559

**Published:** 2022-08-17

**Authors:** Ling Mei, Yan Xu, Qingtong Shi, Chen Wu

**Affiliations:** ^1^Operating Room, The Affiliated Hospital of Yangzhou University, No. 368 Hanjiang Middle Road, Yangzhou, Jiangsu, China; ^2^Department of Thoracic Surgery, The Affiliated Hospital of Yangzhou University, No. 368 Hanjiang Middle Road, Yangzhou, Jiangsu, China

## Abstract

**Objective:**

To explore the application effect and prognostic benefits of whole-course high-quality nursing in lung cancer patients after surgery.

**Methods:**

Sixty patients with lung cancer who underwent surgical treatment in the Department of Respiratory Medicine from April 2020 to July 2021 were recruited and assigned to receive either conventional nursing (control group) or whole-course high-quality nursing (intervention group) using the random number table method, with 30 cases in each group. Outcome measures included self-rating anxiety scale (SAS) scores, self-rating depression scale (SDS) scores, nursing compliance, patient satisfaction, complications, and patient prognosis.

**Results:**

Patients receiving whole-course high-quality nursing showed significantly lower SAS and SDS scores versus those given conventional nursing (*P* < 0.05). Whole-course high-quality nursing resulted in higher patient compliance versus conventional nursing (*P* < 0.05). Patients in the intervention group were more satisfied with the nursing compared with those in the control group (*P* < 0.05). Whole-course high-quality nursing resulted in a lower incidence of complications, postoperative recurrence, and mortality versus conventional nursing (*P* < 0.05).

**Conclusion:**

Whole-course high-quality nursing alleviates the negative emotions of patients after lung cancer surgery, enhances patient compliance and satisfaction, and reduces the incidence of postoperative relapse and complications, which demonstrates great potential for clinical promotion.

## 1. Introduction

Lung cancer is a common malignant tumor with high clinical morbidity and mortality [1]. Due to the insidiousness of early symptoms, the disease may have progressed into the advanced stage by the time of diagnosis, resulting in poor patient prognosis [2]. Surgery is the mainstay of treatment for lung cancer with established effectiveness, but its invasiveness is associated with negative psychological responses of patients, compromising postoperative recovery [3]. Over the past few decades, the treatment of lung cancer has become increasingly precise and diverse, with chemotherapy being widely used in clinical practice. However, chemotherapy may cause collateral damage to the adjacent tissues during treatment, and the most common adverse reactions are digestive tract reactions, bone marrow suppression, and liver function impairment [4]. In view of the shortcomings of chemotherapy, traditional Chinese medicine (TCM), such as acupuncture, TCM herbal compression, and herbal decoction, is encouraged as adjuvant therapy to reduce toxicity of chemotherapy drugs and enhance treatment efficacy [5].

Wang et al. showed that good perioperative nursing might boost postoperative recovery of patients and improve prognosis [6]. Nonetheless, conventional nursing fails to alleviate the patients' adverse emotions and leads to compromised treatment efficacy [7]. The whole-course high-quality nursing is a patient-oriented nursing modality that provides patients with physical and psychological care [8]. Nevertheless, there is dearth of reports on the application of whole-course high-quality nursing in lung cancer patients undergoing surgical treatment [9]. To this end, this study explored the application effect and prognostic benefits of whole-course high-quality nursing in lung cancer patients after surgery to provide relevant references for clinical practice.

## 2. Materials and Methods

### 2.1. Baseline Data

The eligible patients were assigned to a control group (*n* = 30) or intervention group (*n* = 30).

The medical ethics committee has approved this study (no. AHYZ-9597), and all patients and their families signed informed consent.

### 2.2. Inclusion and Exclusion Criteria

#### 2.2.1. Inclusion Criteria

1. Patients were clinically diagnosed with lung cancer
2. Patients underwent surgical treatment in our hospital
3. Patients voluntarily agreed to cooperate with this study

#### 2.2.2. Exclusion Criteria

1. Patients with severe other organ diseases
2. Patients with contraindications
3. Patients with mental abnormalities
4. Patients who were unconscious or unable to cooperate with this study reasonably

### 2.3. Methods

#### 2.3.1. Patients in the Control Group Received Conventional Nursing

The nursing staff provided patients with basic nursing measures such as health education, medication guidance, dietary guidance, and life care. Patients with advanced lung cancer were given dietary plans, with light and high nutrition as the mainstay. In daily care, the nursing staff helped the patients to turn over or change their positions on the bed, massaged their limbs, and performed passive activities. Moreover, analgesic drugs were administered when necessary. Daily instructions such as dietary guidance, exercise instruction, and self-care instructions were provided through regular telephone follow-ups after discharge.

#### 2.3.2. Patients in the Intervention Group Received Whole-Course High-Quality Nursing

*(1) Environmental Nursing*. The humidity and temperature of the operating room were adjusted accordingly to maintain the physical and psychological comfort of the patients, and the nursing staff communicated with the patients after entering the operating room to alleviate their psychological pressure.

*(2) Preoperative Nursing.*

1. The nursing staff carefully assessed the patient's condition to formulate a reasonable nursing plan.
2. The patients were given health education, such as disease knowledge, treatment procedures, and surgery precautions, to enhance their disease awareness and enhance their treatment compliance.
3. The nursing staff provided patients with psychological counseling to mitigate their negative emotions.
4. The patients were also given dietary guidance and assistance in terms of self-care and hospital examinations.
5. The nursing staff communicated with the patients to offer them psychological support, so as to enhance their treatment confidence and compliance [10].

*(3) Intraoperative Nursing.*

  (1) The nursing staff comforted the patients before anesthesia
  (2) The vital signs of the patients were closely monitored by the nursing staff [11]

*(4) Postoperative Nursing.*

1. The patients were given analgesics when necessary
2. The patients were given tailored dietary protocols to promote postoperative recovery
3. After recovery from anesthesia, the patient may experience anxiety, irritability, and other emotions. If the patient's mood fluctuates significantly, the nursing staff should use the restraint belt to avoid the accidental extubation and falling of the patient.
4. The nursing staff should pay attention to preventing complications such as pressure ulcers and lower extremity deep vein thrombosis. Complications, if any, were promptly managed.
5. During the bandage change, the nursing staff should check for any signs of infection and the color and amount of any drainage
6. The patients were informed of the surgery outcome and postoperative cautions after full recovery of patients from anesthesia [12]
7. Patients in both groups were followed up for two years after surgery, with one telephone follow-up every month and one home follow-up every year.

### 2.4. Observation Indicators

1. Self-rating anxiety scale (SAS) and self-rating depression scale (SDS) scores [13, 14]: SAS was used to evaluate the anxiety of patients, with a score ranging from 0 to 100 points and a cutoff value of 50 points, of which 50 to 59 indicates mild anxiety, 60–69 indicates moderate anxiety, and 69 or more indicates severe anxiety. SDS was used to evaluate the degree of depression of the patients, with a score of 0–100 and a cutoff value of 53 points, of which 53–62 indicates mild depression, 63–72 indicates moderate depression, and 73 or above indicates severe depression.
2. Nursing compliance: the nursing compliance was assessed with a full score of 100 points, with ≥90 for good compliance, 70–89 for general compliance, <70 for poor compliance. Compliance=(good + general)/total cases × 100%.
3. Nursing satisfaction: the “nursing satisfaction questionnaire” made by the hospital was used. There are 20 questions in this questionnaire, and the total score is 100 points, with <70 points for dissatisfied, 70–89 points for satisfied, and ≥90 points for very satisfied. Satisfaction = (very satisfied + satisfied)/total number of cases × 100%.
4. Complications: postoperative complications include infection, bleeding, pressure ulcers, and fever.
5. Prognosis: The disease recurrence and mortality of the patients were recorded.

### 2.5. Statistical Methods

Statistical analysis of the data was done using the SPSS20.0 software. The measurement data were expressed as (mean ± standard deviation) and analyzed using the *t*-test. The counting data were expressed as the number of cases (rate) and subject to the X^2^ test. *P* < 0.05 indicates the presence of statistical significance. GraphPad Prism 8 was selected as the mapping software.

## 3. Results

### 3.1. Patient Characteristics

In the control group, there were 21 males and 9 females, aged 25 to 61 (48.23 ± 8.15) years, with 17 cases of tumor, node, metastasis (TNM) stage I, 9 cases of stage IIa, and 4 cases of stage IIIa. In the intervention group, there were 20 males and 10 females, aged 24 to 62 (48.34 ± 8.23) years, with 19 cases of TNM stage I, 7 cases of stage IIa, and 4 cases of stage IIIa. There was no significant difference in general data between the two groups (*P* > 0.05), as shown in Table 1.

### 3.2. SAS and SDS Scores

Patients receiving whole-course high-quality nursing showed significantly lower SAS and SDS scores (45.33 ± 4.21, 46.56 ± 4.87) versus those given conventional nursing (54.74 ± 5.15, 55.28 ± 5.31) (*P* < 0.05), as shown in Table 2.

### 3.3. Nursing Compliance

Whole-course high-quality nursing resulted in higher patient compliance (97%) versus conventional nursing (70%) (*P* < 0.05), as shown in Table 3.

### 3.4. Nursing Satisfaction

More patients were satisfied with the nursing method in the intervention group (100%) than in the control group (63%) (*P* < 0.05), as shown in Table 4.

### 3.5. Complications

The incidence of complications in the intervention group (5%) was significantly lower than in the control group (28%) (*P* < 0.05), as shown in Table 5.

### 3.6. Prognosis

Patients receiving whole-course high-quality nursing had a lower recurrence rate and mortality at 1 and 2 years after surgery than those given conventional nursing (*P* < 0.05), as shown in Table 6.

## 4. Discussion

Lung cancer is associated with high clinical mortality and morbidity. Lung cancer includes non-small-cell lung cancer (NSCLC) and small-cell lung cancer, of which NSCLC accounts for more than 85% [15]. In the clinical research of lung cancer over the years, the treatment of lung cancer has become more and more precise and diversified, and chemotherapy is widely used in clinical practice [16]. The prevalence of lung cancer in China has been growing year after year as people's lifestyles and dietary habits have changed [17]. Due to the insidiousness of early symptoms, the disease may have progressed into the advanced stage by the time of diagnosis, resulting in poor patient prognosis [18]. Current treatments for lung cancer include surgery, chemotherapy, and radiotherapy, and TCM treatment is also effective as adjuvant therapy to enhance the treatment efficiency and reduce adverse events. Surgery is the treatment of choice for early lung cancer with recognized effectiveness [19]. However, Li[20] stated that the invasive nature of surgery is associated with a cascade of postoperative adverse reactions, which compromises the treatment outcomes and prognosis of patients [21]. In addition, Wang [22] noted that most patients are unaware of the disease and its treatment, which leads to negative emotions such as anxiety and depression during treatment. The research by Wang et al. [23] demonstrated that perioperative nursing plays an important role in enhancing the postoperative recovery of patients, alleviating their negative emotions and complications, and improving their prognosis. In whole-process high-quality nursing, the patients are provided with both physical and psychological care perioperatively. The whole-process high-quality nursing provides patients with physiological and psychological nursing rather than focusing solely on medical care during hospitalization [24].

The results of the present study showed that patients receiving whole-process high-quality nursing had lower SAS and SDS scores, a lower incidence of complications, and higher satisfaction than those given conventional nursing. The reason may be that during whole-process high-quality nursing, targeted psychological counseling increased the patients' treatment confidence and reduced their anxiety and depression, which improved their nursing compliance and satisfaction and reduced the incidence of postoperative complications [25]. Research by Li et al. [26] has shown that negative emotions resulted in a 13% reduction in lung cancer patients' survival rates, which suggested the role of effective psychological intervention in the postoperative nursing of patients. Furthermore, whole-process high-quality nursing also contributes to enhancing the immune function and treatment efficiency of patients, as evidenced by the lower recurrence rate and mortality rate of patients in the intervention group at 1 year and 2 years after surgery than those in the control group. The reason may be that whole-process high-quality nursing effectively regulates the psychological status of lung cancer patients and prevents postoperative complications, which facilitates the recovery of the immunity of patients, thereby prolonging patient survival [27].

## 5. Conclusion

Whole-course high-quality nursing alleviates the negative emotions of patients after lung cancer surgery, enhances patient compliance and satisfaction, and reduces the incidence of postoperative relapse and complications, which demonstrates great potential for clinical promotion.

## Figures and Tables

**Table 1:** Patient characteristics.

	Control group (*n* = 30)	Intervention group (*n* = 30)	*t*/*x*^*2*^	*P* value
Gender			0.077	0.781
Male	21	20		
Female	9	10		
Age	25–61	24–62		
Average age	48.23 ± 8.15	48.34 ± 8.23	−0.052	0.959
TNM stages			0.361	0.548
Stage I	17	19		
Stage IIa	9	7		
Stage IIIa	4	4		

**Table 2:** Comparison between SAS and SDS scores $\left(\bar{x}\pm s\right)$.

Groups	Number of patients	SAS score		SDS score	
		Before nursing	After nursing	Before nursing	After nursing
Control group	30	64.32 ± 5.63	54.74 ± 5.15	64.17 ± 6.34	55.28 ± 5.31
Intervention group	30	65.23 ± 4.84	45.33 ± 4.21	63.82 ± 6.19	46.56 ± 4.87
*t*	—	-0.671	7.748	0.216	6.629
*P*	—	0.505	＜0.001	0.83	＜0.001

**Table 3:** Comparison of nursing compliance (*n* (%)).

Groups	Patients	Good	Satisfactory	Poor	Overall compliance rate
Control group	30	9	12	9	21 (70%)
Intervention group	30	18	11	1	29 (97%)
*x* ^*2*^	—	—	—	—	7.68
*P*	—	—	—	—	0.006

**Table 4:** Comparison of nursing satisfaction (*n* (%)).

Groups	Patients	Very satisfied	Satisfied	Unsatisfied	Overall satisfaction rate
Control group	30	10	9	11	19 (63%)
Intervention group	30	22	8	0	30 (100%)
*x* ^*2*^	—	—	—	—	13.469
*P*	—	—	—	—	＜0.001

**Table 5:** Comparison of complications (*n* (%)).

Groups	Patients	Infections	Bleeding	Pressure ulcers	Fever	Overall complication rate
Control group	30	4	1	2	4	11 (28%)
Intervention group	30	1	0	0	1	2 (5%)
*x* ^*2*^	—	—	—	—	—	7.44
*P*	—	—	—	—	—	0.006

**Table 6:** Comparison of prognosis (*n* (%)).

Groups	Patients	First year		Second year	
		Recurrence rate (%)	Death rate (%)	Recurrence rate (%)	Death rate (%)
Control group	30	6 (20%)	4 (13%)	11 (37%)	7 (23%)
Intervention group	30	2 (7%)	0 (0%)	5 (17%)	1 (3%)
*x* ^*2*^	—	7.236	13.904	10.147	17.683
*P*	—	0.007	＜0.001	0.001	＜0.001

## Data Availability

No data were used to support this study.
